The article "Blockchain and K-Means Algorithm for Edge AI Computing" was retracted in 2023. Reasons: unreliable results or conclusions; concerns about the data; concerns about the results or conclusions; concerns about the peer review.

# Blockchain and K-Means Algorithm for Edge AI Computing

**DOI:** 10.1155/2022/1153208

**Published:** 2022-05-29

**Authors:** Xiaotian Qiu, Dengfeng Yao, Xinchen Kang, Abudukelimu Abulizi

**Affiliations:** ^1^Beijing Key Laboratory of Information Service Engineering, Beijing Union University, Beijing 100101, China; ^2^School of Computer Science and Engineering, University of Electronic Science and Technology of China, Chengdu 611731, Sichuan, China; ^3^Department of Information Management, Xinjiang University of Finance and Economics, Urumqi 830012, Xinjiang, China

## Abstract

The current development of blockchain, technically speaking, still faces many key problems such as efficiency and scalability issues, and any distributed system faces the problem of how to balance consistency, availability, and fault tolerance need to be solved urgently. The advantage of blockchain is decentralization, and the most important thing in a decentralized system is how to make nodes reach a consensus quickly. This research mainly discusses the blockchain and K-means algorithm for edge AI computing. The natural pan-central distributed trustworthiness of blockchain provides new ideas for designing the framework and paradigm of edge AI computing. In edge AI computing, multiple devices running AI algorithms are scattered across the edge network. When it comes to decentralized management, blockchain is the underlying technology of the Bitcoin system. Due to its characteristics of immutability, traceability, and consensus mechanism of transaction data storage, it has recently received extensive attention. Blockchain technology is essentially a public ledger. This is done by recording data related to trust management to this ledger. To collaboratively complete artificial intelligence computing tasks or jointly make intelligent group decisions, frequent communication is required between these devices. By integrating idle computing resources in an area, a distributed edge computing platform is formed. Users obtain benefits by sharing their computing resources, and nodes in need complete computing tasks through the shared platform. In view of the identity security problems faced in the sharing process, this article introduces blockchain technology to realize the trust between users. All participants must register a secure identity in the blockchain network and conduct transactions in this security system. A K-means algorithm suitable for edge environments is proposed to identify different degradation stages of equipment operation reflected by multiple types of data. Based on the prediction of the fault state for a single type of data, the algorithm uses the historical data of multiple types of data together with the prediction data to predict the fault stage. During the research process, the average optimization energy consumption of K-means algorithm is 14.6% lower than that of GA. On the basis of designing a resource allocation scheme based on blockchain, the problem of how the participants can realize reliable resource use according to the recorded data on the chain is studied. The article implements the verification of the legality of the use of blockchain resources. In addition, a control node is introduced to master the global real-time information of the network to provide data support for the user's choice.

The article "Blockchain and K-Means Algorithm for Edge AI Computing" was retracted in 2023. Reasons: unreliable results or conclusions; concerns about the data; concerns about the results or conclusions; concerns about the peer review.

## 1. Introduction

Under certain growth conditions, the quantum dots in the multilayer quantum dot structure can also be ordered in the lateral direction. Thus, a chain-like quantum dot structure is formed, here we call it a quantum chain. Since the interval between quantum dots on the same chain can be very small, resulting in lateral coupling between carriers, it exhibits unique optical properties. The proof of stake is represented by the quantum chain, although the transaction confirmation speed is very fast, there is a problem with the concentration of rights. The efficiency of the consensus mechanism greatly affects the speed of blockchain transactions and block confirmation, and it cannot be well applied to the consortium chain scenario. Consensus mechanisms such as Proof of Work and Proof of Stake have the above performance bottlenecks in the application of consortium chains. Therefore, in the consortium chain scenario, it is necessary to design an efficient consensus algorithm to meet the requirements of high throughput and low latency. Proof of Stake, or POS for short, is also called a consensus protocol. The upgraded consensus mechanism of PoW is similar to depositing assets in a bank. The bank will distribute the corresponding income according to the amount and time of digital assets it hold. PoS determines your probability of obtaining bookkeeping rights by evaluating the number and duration of tokens it hold. This is similar to the dividend system of stocks, and those who hold relatively more equity can get more dividends.

This article takes blockchain technology as the research background, and the blockchain has aroused great repercussions since the birth of Bitcoin. Block proposes a decentralized, trustless financial system implementation. Inspired by Bitcoin, Ethereum proposes a decentralized application combined with smart contracts. The research further designs and implements a simulation experiment scheme based on the existing Ethereum blockchain platform. Using the smart contracts supported by Ethereum, the business logic of resource provision and resource request information release functions is written into the contract in the form of code.

The article "Blockchain and K-Means Algorithm for Edge AI Computing" was retracted in 2023. Reasons: unreliable results or conclusions; concerns about the data; concerns about the results or conclusions; concerns about the peer review.

For the problem of decentralized resource provision and resource request release, the peer-to-peer network and self-authentication encryption technology commonly used in blockchain technology are adopted. It realizes the provision of decentralized trusted resources and the release of resource requests between edge nodes. The K-means algorithm is an algorithm based on initialized cluster centers. The similarity between each data is evaluated by calculating the Euclidean distance, and the object data is divided into different clusters according to the calculated similarity. After the division, the data similarity in the same cluster is relatively high, and the data similarity between different clusters is relatively low. After each division is completed, the center of each cluster needs to be recalculated. It then continues to perform the above process iteratively until all data partitioning is complete. With the development of the Internet of Things, autonomous edge computing requires reliable and secure data communication without relying on centralized cloud servers. It uses blockchain to achieve consensus on various transactions and ensure trust between edge entities.

## 2. Related Work

Artificial intelligence is a branch of computer science. It attempts to understand the essence of intelligence and produce a new intelligent machine that can respond in a similar way to human intelligence. Research in this area includes robotics, language recognition, image recognition, natural language processing, and expert systems. Since the birth of artificial intelligence, theory and technology have become more and more mature, and the application field has also expanded. Hardware architectures and platforms continue to maintain rapid development to meet the requirements of computationally intensive machine learning models. The boom in dedicated accelerators is contributing to further improvements in throughput and energy efficiency. Therefore, driven by breakthroughs in machine learning and upgrades in hardware architecture, artificial intelligence is continuing to achieve impressive achievements. Zhang et al. believe that clustering is a common technique for multimedia organization, analysis, and retrieval. However, most multimedia clustering methods have difficulty in capturing high-order nonlinear correlations on multimodal features, resulting in low clustering accuracy. Furthermore, they cannot extract features from multimedia data with missing values. As a result, it is impossible to cluster the incomplete multimedia data ubiquitous in practical applications. He proposed a high-order possible C-means algorithm (HOPCM) for clustering incomplete multimedia data. HOPCM improves the basic autoencoder model for learning features of multimedia data with missing values. Furthermore, HOPCM uses tensor distance instead of Euclidean distance as the distance metric to capture as much of the unknown high-dimensional distribution of multimedia data as possible. He conducts extensive experiments on three representative multimedia datasets such as NUS-WIDE, CUAVE, and SNAE [1]. Kumar et al. believe that data clustering is an important data mining technique for creating groups of objects (clusters). It makes objects in one cluster very similar and very different in different clusters. The Fuzzy c-Means (FCM) algorithm is a popular data clustering method that operates on fuzzy memberships between data points and cluster centers. However, it has the potential to converge to a local minimum. The Artificial Bee Colony (ABC) algorithm is a bee colony-based algorithm. It is inspired by the intelligent foraging behavior of bees. To take full advantage of the advantages of these two algorithms, he proposed a hybrid algorithm based on the improved ABC and FCM algorithms (IABCFCM) [2]. Alsmadi believes that early diagnosis of jaw tumors is very important to improve their prognosis. Differential diagnoses can be made using X-ray images. Therefore, accurate and fully automatic image segmentation of jaw lesions is a challenging and necessary task. The aim of his work is to develop a novel, fully automatic, and efficient method for jaw lesions in panoramic X-ray image segmentation. The hybrid fuzzy C-means method was used to segment jaw images and detect jaw lesion regions in panoramic X-ray images, which may be helpful in diagnosing jaw lesions. Area error metrics are used to evaluate the performance and efficiency of the proposed method from different aspects. He performed specificity, sensitivity, and similarity analyses to assess the robustness of the proposed method. He compares the proposed method with the hybrid firefly algorithm with fuzzy C-means and the artificial bee colony with fuzzy C-means algorithm [3]. Yang et al. believe that the traditional K-means algorithm has been widely used as a simple and efficient clustering method. However, the performance of this algorithm is highly dependent on the choice of initial cluster centers. Therefore, the method used to select the initial cluster centers is extremely important. He redefines the density of points based on the number of adjacent points and the distance between points and adjacent points. Furthermore, he defines a new distance metric that takes into account both Euclidean distance and density. On this basis, he proposed an initial cluster center selection algorithm that can dynamically adjust the weight parameters. Furthermore, he proposes a new internal clustering validation metric namely, the Neighborhood-based Cluster Validation Index (CVN), which can be used to select the optimal result among multiple clustering results. His proposed algorithm outperforms existing initialization methods on real-world datasets. He also demonstrated the adaptability of the algorithm to datasets with various characteristics [4]. Qin et al. focus on developing distributed k-means algorithm and distributed fuzzy C-means algorithm for wireless sensor networks (WSN) equipped with sensors at each node. The underlying topology of WSN should be strongly connected. He uses the consensus algorithm in the multi-agent consensus theory to exchange the measurement information of the sensors in the WSN. To obtain a faster convergence speed and a higher probability of obtaining the global optimum, he first proposed a distributed k-means algorithm. He finds the initial centroids before executing the distributed k-means algorithm and the distributed fuzzy C-means algorithm. His proposed distributed k-means algorithm is able to divide the data observed by nodes into metrically related groups with within-group distances and large-group distances. The proposed distributed fuzzy C-means algorithm is able to divide the data observed by nodes into different measurement-related groups [5]. Cabria and Gondra argue that cyber-physical systems typically consist of a large number of spatially distributed autonomous sensors. These sensors monitor physical conditions and communicate with key locations. He considers the problem of locating mobile storage facilities in a recycling network consisting of two types of nodes such as collection points (neighborhood recycling bins) and mobile storage centers, and the problem of finding the optimal number of storage centers. Sensors at the collection point monitor the fill level and transmit it to the main location where the collection point gathers. He proposed a variant of K-means, latent K-means. It assigns each cluster to a storage center and balances the load of the storage centers. For a fixed number of storage centers, it can minimize the total network cost [6]. One of the things that people are questioning about AI is that it's like a black box. The results are difficult to explain theoretically, and blockchain is known for securely and accurately recording transactions without tampering in peer-to-peer decentralized scenarios. Recording the intermediate results and decision-making process of artificial intelligence on the blockchain can increase its transparency. It is conducive to public acceptance and trust in decision-making, and it is also convenient for relevant personnel to audit. At the same time, in the scenario of edge artificial intelligence computing, which may involve multiparty intelligent joint decision-making. Edge computing is a complementary solution to cloud computing. It extends the functions of cloud computing to the edge of the network closer to the source of data generation to reduce the burden of network transmission. At the same time, it is more suitable for some applications.

The article "Blockchain and K-Means Algorithm for Edge AI Computing" was retracted in 2023. Reasons: unreliable results or conclusions; concerns about the data; concerns about the results or conclusions; concerns about the peer review.

## 3. Blockchain and K-Means Algorithm for Edge AI Computing

### 3.1. System Model

The system model is shown in Figure 1. The network describes a system model in which a group of users participating in a consensus competition obtains computing power from a group of edge servers. To increase the probability of winning in the consensus competition, the intelligent terminal *i* obtains computing resources from the edge server *k* and pays the corresponding fees. Here, *x*_*i*_^*k*^ is used to represent the computing power obtained by the smart terminal *i* from the edge server *k*, and *x*_*i*_^loc^ is used to represent the computing power of the smart terminal *i* itself. Edge computing is a type of distributed computing technology. It is the general trend to combine the method of data processing near the terminal of the IoT device and the blockchain. However, many issues of security, uneven distribution of computing resources, and supervision need to be addressed.

In this model, the total computing power *i* of the intelligent terminal *i* consists of the computing power obtained from the edge server and the local computing power. It is represented by the following formula [7]:

(1) $$\begin{array}{c} \chi =x_{i}^{\text{loc}}+\sum_{k\in \xi }x_{i}^{k}. \end{array}$$

The ratio of the computing power of the smart terminal *i* to the computing power of all smart terminals is represented by *i* [8]:

(2) $$\begin{array}{c} \alpha =\frac{\beta }{\sum \beta }=\frac{x_{i}^{\text{loc}}+\sum_{k\in \varsigma }x_{i}^{k}}{\sum x_{i}^{\text{loc}}+\sum_{i\in I}\sum_{k\in \varsigma }x_{i}^{k}}. \end{array}$$

The success probability P of the intelligent terminal *i* winning in the consensus competition can be modeled as a random variable as follows [9]:

(3) $$\begin{array}{c} P\left(\alpha ,t\right)=\alpha \left(1-P\left(t\right)\right). \end{array}$$

Among them, *t*_*i*_ represents the block size recorded by smart terminal *i* [10].

(4) $$\begin{array}{c} P\left(t\right)=1-e^{-\lambda t}, \end{array}$$

*P*(*t*) is the abandonment probability. The role of *P*(*t*) is explained as follows. After solving the PoW (proof of work), the smart terminal *i* needs to broadcast the obtained result to other smart terminals to reach a consensus. Due to the delay in broadcasting the calculation results to other nodes, it is possible that the first intelligent terminal *i* that calculates the result of the proof-of-work problem cannot be the first node to reach a consensus. This probability can be represented by the abandonment probability of *P*(*t*).

The article "Blockchain and K-Means Algorithm for Edge AI Computing" was retracted in 2023. Reasons: unreliable results or conclusions; concerns about the data; concerns about the results or conclusions; concerns about the peer review.

The intelligent terminal *i* wins the right to record the block and obtains the corresponding income can be expressed as follows [11]:

(5) $$\begin{array}{c} m_{i}=\left(R+r\right)P\left(\alpha ,t\right)-\sum px_{i}^{k}. \end{array}$$

The parameter *p* indicates the unit price of the computing power provided by the edge server *k* to the intelligent terminal *i*.

### 3.2. Multiuser-Multi-Edge Server Scenario Problem Modeling

Next, we study the multi-edge server scenario and focus on solving the sub-problem (TRO-Sub) and the top-level problem (TRO-Top). The problem (TRO-ES) is a non-convex optimization problem that is generally difficult to solve. To this end, vertical decomposition is adopted again here, and an auxiliary variable *v*_*i*_ is introduced to represent the computing power obtained by intelligent terminal *i* from all edge servers, namely [12]:

(6) $$\begin{array}{c} v_{i}=\sum_{i\in k}x_{i}^{k}. \end{array}$$

First, assuming that the value of {*v*_*i*_} is given in advance, the goal is to solve the sub-problem as follows:

(7) $$\begin{array}{c} H_{\left\{v_{i}\right\}}^{\text{sub}}=\max\sum \ln\left(\left(R+rt\right)\sum_{i=1}\chi \frac{x+v}{\lambda \left(x+v\right)}e+\sum_{i=1}\pi px\right),\\ \theta =\sum_{\text{k}=1}^{m}x_{i}^{k}v. \end{array}$$

After solving the sub-problem (TRO-Sub) and obtaining *H*_{*v*_*i*_}_^sub^ (corresponding to the given {*v*_*i*_}), proceed to solve the top-level problem as follows [13]:

(8) $$\begin{array}{c} {\left(\text{TRO}-\text{Top}\right)}_{\max}=\max H_{\left\{v_{i}\right\}}^{\text{sub}},\\ 0\leq {\text{v}}_{\text{i}}\leq Q,\;\forall i\in I. \end{array}$$

Among them [14],

(9) $$\begin{array}{c} Q=\sum_{k\in K}C^{k,\text{tot}}. \end{array}$$

### 3.3. Total Energy Consumption of Data Processing

The blockchain system consists of a data layer, network layer, consensus layer, incentive layer, contract layer, and application layer. In the process of data processing, the total energy consumption of the edge blockchain must be minimized for maximum benefit. The total energy consumption mainly includes the data storage energy consumption and data transmission energy consumption between the edge computing server and the blockchain. The total energy consumption can be expressed as [15]

(10) $$\begin{array}{c} C_{c}=C_{n}+C_{nk}^{t}. \end{array}$$

Considering the benefit and load balancing of the edge computing system based on blockchain, the total energy consumption *C*_*c*_ of block data processing is [16]

(11) $$\begin{array}{c} C_{c}=C_{n}+C_{nk}^{t}=k\sum_{i=1}^{k}d\left(\alpha +\beta s\right). \end{array}$$

Considering the calculation of data storage energy consumption and data transmission energy consumption, the total energy consumption of data processing can be minimized only when the appropriate *α* and *β* are found. So the total energy consumption objective function of block data processing is [17]

(12) $$\begin{array}{c} \min f=\min k\sum_{t=1}^{k}d\left(\alpha +\beta s\right),\left(\alpha ,\beta \in \left(0,1\right)\right). \end{array}$$

The article "Blockchain and K-Means Algorithm for Edge AI Computing" was retracted in 2023. Reasons: unreliable results or conclusions; concerns about the data; concerns about the results or conclusions; concerns about the peer review.

### 3.4. Overall Net Income Value of Users

The underlying problem (TRO-Sub) after {*v*_*i*_} is given is a convex optimization problem. Therefore, the joint optimization variable *λ*^*k*^ is introduced again here to relax the constraints on ESk and obtain the corresponding Lagrangian function [18]:

(13) $$\begin{array}{c} L\left(\left\{x_{i}^{k}\right\},\left\{\lambda_{i}^{k}\right\}\right)=\sum_{i\in I}\ln\left[\left(R+t\right)M-px+\lambda \left(C^{k,\text{tot}}-\sum_{i\in I}x_{i}^{k}\right)\right]. \end{array}$$

Among them, the parameter *M* represents the proportion of the computing power of the intelligent terminal *i* in a group of intelligent terminals. The expression is [19]

(14) $$\begin{array}{c} M=\frac{x_{i}^{\text{loc}}+v_{i}}{\sum \left(x_{i}^{\text{loc}}+v_{i}\right)}e^{-\lambda t}. \end{array}$$

It can be found that it can be separated as follows [20]:

(15) $$\begin{array}{c} L\left(\left\{x_{i}^{k}\right\},\left\{\lambda_{i}^{k}\right\}\right)=\sum_{i\in I}L\sum_{\mu =1}\chi \left[px+L\left({\left\{x_{i}^{k}\right\}}_{\forall k\in K},{\left\{\lambda_{i}^{k}\right\}}_{\forall k\in K}\right)\right]+\sum_{k\in K}C^{k,\text{tot}}. \end{array}$$

The Lagrangian formula corresponding to each smart terminal *i* is as follows [21]:

(16) $$\begin{array}{c} L_{i}\left({\left\{x_{i}^{k}\right\}}_{\forall k\in K},{\left\{\lambda_{i}^{k}\right\}}_{\forall k\in K}\right)=\ln\sum_{i\in I}\left(R+rt\right)\left[px+M\right]+\sum_{k\in K}x_{i}^{k}\lambda . \end{array}$$

Here, the local optimization problem of each intelligent terminal *i* is formulated as follows:

(17) $$\begin{array}{c} \left\{x_{i}^{k}\right\}=\arg\max\;\ln\left(\left(R+t\right)M-\sum px\right)-\sum p\lambda . \end{array}$$

To further determine the optimal value of {*λ*_*i*_^*k*^}_∀*k*∈*K*_ (i.e., the optimal solution to the dual problem), the following sub-gradient method [22] is used in this study:

(18) $$\begin{array}{c} \lambda^{k}=\max\left\{\lambda^{k}-\varepsilon \left(C^{k,tot}-\sum_{i\in I}x_{i}^{k}\right),0\right\}, \end{array}$$

where *ε* is the step size of the double update.

The article "Blockchain and K-Means Algorithm for Edge AI Computing" was retracted in 2023. Reasons: unreliable results or conclusions; concerns about the data; concerns about the results or conclusions; concerns about the peer review.

### 3.5. Energy Consumption Optimization of Edge Blockchain Based on K-Means Algorithm

In the algorithm proposed in this study, the setting of initializing the cluster center is the same as that of the K-means algorithm, that is, it is set randomly. Then, based on the initialized cluster center, the similarity between each data is evaluated by the calculation of Euclidean distance. It divides the object data into different clusters according to the level of similarity. Factors such as the order of data in this algorithm will not affect the results of clustering. Therefore, the algorithm does not consider the order of the data and only classifies it according to the characteristics of the data. In this algorithm, due to the different characteristics of data in different degradation stages, the similarity between data in the same stage is much higher than that between data in different stages. Therefore, if there are different stages of data in the classified data, the algorithm can effectively distinguish the degraded data of different stages. In this algorithm, after the first division is completed, the number of remaining cluster centers is determined according to the results. The cluster centers that are not reserved will be initialized to the newly collected data in the next classification so that the emergence of new stages can be better identified. In this study, the K-means algorithm is used as the edge intelligence to divide the degradation stage. The threshold for the division is relatively low, so the number of iterations is used as the convergence condition of the algorithm.

First, the terminal device sends a request to the edge server to store data in the blockchain, and then the edge server queries whether there are free blocks in the blockchain. If there are free blocks, the data storage is distributed in the blockchain. Otherwise, it denies the data storage service. Finally, the K-means algorithm is used iteratively to find the position of the optimal particle. Even *C*_*C*_ reaches the minimum of *α* and *β*, and gets the minimum energy consumption of *C*_*C*_.

It initializes the dataset *X*. The dataset is composed of *n* data collected, namely, [23]

(19) $$\begin{array}{c} X=\left\{X_{1},X_{2},X_{3},\text{…},X_{\text{n}}\right\}. \end{array}$$

Its request batching latency refers to the time to batch requests:

(20) $$\begin{array}{c} l_{b}=\frac{h\Delta t}{R_{is}}, \end{array}$$

where *R*_*is*_ is the average number of machine learning requests processed during *s* by the last instance of version *i* on dataset Δt.

The article "Blockchain and K-Means Algorithm for Edge AI Computing" was retracted in 2023. Reasons: unreliable results or conclusions; concerns about the data; concerns about the results or conclusions; concerns about the peer review.

Each data object is *m*-dimensional data:

(21) $$\begin{array}{c} X_{1}=\left\{X_{1},X_{2},X_{3},\text{…},X_{\text{m}}\right\}. \end{array}$$

Computing the sum of squares of the distances from each data object in cluster *c*_*i*_ to the center *u* of the cluster can be expressed by the following formula [24]:

(22) $$\begin{array}{c} J\left(c_{k}\right)={\sum_{x_{i}\in c_{i}}\left\|x_{i}-u_{k}\right\|}^{2}. \end{array}$$

It redetermines cluster centers and clusters until the sum of the squares of the distances between each data object and the corresponding cluster center reaches a minimum. The objective function formula of its algorithm is [25]

(23) $$\begin{array}{c} J\left(C\right)=\sum_{k=1}^{K}J\left(C_{k}\right)={\sum_{k=1}\sum_{k=1}\left\|x_{i}-u_{i}\right\|}^{2}{\sum_{k=1}\sum_{k=1}\lambda \left\|x_{i}-u_{i}\right\|}^{2}. \end{array}$$

Among them, if *x*_*i*_ ≤ *u*_*i*_, then *λ*=1, otherwise *λ*=0.

### 3.6. BACombo (Bandwidth—Aware Combo) System Implementation

As a decentralized federated learning system, each node is trained locally. At the same time, the aggregation of the global model is also performed. But at the same time, it still needs the participation of a coordinator server, this coordinator server only maintains the system metadata. Its main job is to initialize the model parameters of each node with the same values and transmit them to all participating nodes before training starts. At the same time, the server has the information of all nodes, and also broadcasts the node list when initializing the parameters.

1. Local update: the learning process starts with the node updating the model using the local dataset. Nodes take the aggregated results of the last communication round as input to the model and update it using stochastic gradient descent (SGD) on local data. To reduce communication costs, local updates may contain multiple SGD rounds before communicating with other nodes. We denote the communication interval or the number of SGD rounds as *t*, which may take up to several Epochs in a typical federated learning system.
2. Node selection: the node selection part mainly involves two small modules such as bandwidth monitoring and node selection. Each node stores a bandwidth table with all other peer nodes. At the very beginning, this table is initialized to 0. Once a peer node is selected in the communication round, the bandwidth monitoring module will monitor the fragment transmission time. And through the loopback time (RTT) to estimate the available bandwidth of the link. After smoothing the bandwidth value with the bandwidth values recorded in the previous communication rounds, it is stored in the bandwidth table. In the node selection part, each node selects peer nodes in two ways, random selection or greedy selection.
3. Fragment Pull: the node first decides how to partition the model. They don't have to follow the same division rules. But for simplicity, we assume that they divide the model into S shards in the same way. For each shard, a node must choose *R* peers and send pull requests. The request contains a shard description and the node's unique identifier to indicate which part of the model to send and to whom to send the model. Each node must send *S* × *R* shard pull requests to other nodes, whereas BACombo tries to distribute these requests evenly among all nodes to use more links and balance the transfer workload. Therefore, for each request, the target node is randomly selected with no replacement from all other nodes until there are no remaining options. This means that when *S* × *R* < *n*, all shards come from different nodes. Notably, for each communication round, a pull request can even be sent before the local update starts. This way, the target node can send shards as soon as the local model is ready.
4. Sending fragments. The sending process is the dual action of shard pulling. When the node completes the local update, it can send its update result to others. Instead of actively pushing models, nodes schedule model shards only based on received pull requests.
5. Model aggregation. When a node makes model shards available to others, it also receives previously requested shards. The model aggregation phase blocks until all pull requests are satisfied, then the node aggregates the external model shards with the local model and puts the aggregated shards together to rebuild the model. With the aggregated results, the node will go back to the first step and start the next local training. The structure of the BACombo node is shown in Figure 2.

The article "Blockchain and K-Means Algorithm for Edge AI Computing" was retracted in 2023. Reasons: unreliable results or conclusions; concerns about the data; concerns about the results or conclusions; concerns about the peer review.

## 4. Blockchain and K-Means Algorithm Results for Edge AI Computing

To verify the effectiveness of the proposed method for the benefit of the system, MATLAB software is used as the simulation experiment platform. Assuming that there are 10 blocks in the blockchain, the data set information of 10 blocks (blocks 0–9) is shown in Table 1. There are free blocks in the blockchain, so data can be stored. The optimized objective function is used as the fitness function.

To verify the low energy consumption performance of K-means, under the bandwidth of 30 Mbps, and when the number of MEC servers *n* is 10, 50, and 100, respectively, with a simulated annealing (SA) algorithm, the optimization results of Genetic Algorithm (GA), Ant Colony Algorithm (ACO), and K-means algorithm are compared. The minimum energy consumption of the four algorithms is shown in Table 2.

The energy consumption optimization values of various algorithms under different MEC numbers are shown in Figure 3. It can be seen intuitively that with the increase in the number of edge servers, the energy consumption of the four algorithms increases. Under the same MEC server, K-means has the lowest energy consumption. The energy consumption value of the ACO algorithm is second, while the energy consumption value of the GA algorithm and SA algorithm is high and the difference is not big. And the average optimization energy consumption of the K-means algorithm is 14.6% lower than GA, 12.1% lower than SA, and 4.2% lower than ACO.

The iteration times of the four algorithms (GA, SA, ACO, and K-means algorithms) are compared in Table 3.

The iterative process of the four algorithms is shown in Figure 4. With the increase of the MEC scale, the convergence curves of the K-means algorithm are quite different. This shows that the K-means algorithm can adapt to the changes in the MEC server and seek the optimal value in time according to the changes in the number of MECs. However, the iterative curves of GA, SA, and ACO algorithms are not much different, and the optimization process is relatively slow whether in small-scale servers or large-scale servers. The Genetic Algorithm (GA) algorithm is designed and proposed according to the evolution law of organisms in nature. It is a computational model of the biological evolution process that simulates the natural selection and genetic mechanism of biological evolution. It is a process that simulates natural evolution.

To verify the influence of the number of blocks on the energy consumption of data processing under different network bandwidths, when the bandwidth is 30 Mbps, 100 Mbps, 200 Mbps, and 300 Mbps. The changes in the number of blocks and the energy consumption of processing data are shown in Figure 5. As the number of blocks increases, the energy consumption of data processing increases significantly. However, when the data transmission amount is as small as 30 Mbps, the energy consumption gradually becomes stable when the number of blocks is 4. When the network bandwidth is 300 Mbps, the energy consumption changes greatly and tends to be stable when the number of blocks is 8. It shows that in the process of simulation experiment of K-means, the network bandwidth is limited, and the amount of data transmission is limited. By increasing the number of blocks to complete resource storage, the total energy consumption is increased.

The article "Blockchain and K-Means Algorithm for Edge AI Computing" was retracted in 2023. Reasons: unreliable results or conclusions; concerns about the data; concerns about the results or conclusions; concerns about the peer review.

The divided blockchain main chain is 0-2-5-3, and 1-4 is the side chain connected to the node. In a blockchain-based edge computing system, as the number of block nodes in the edge server increases, the blockchain is fragmented. Mainchain and sidechain transactions are distributed and executed in parallel, and each edge block is more efficient in the data processing. The delay comparison of different processing schemes is shown in Figure 6.

According to the specific values, this article makes specific settings for each parameter. Specifically, the block generation rate is set in the simulation (that is, the average generation time of each block is 10 minutes). The block size mined by each smart terminal is set to *t* = 1 Mbit. At the same time, the fixed income of each block in the simulation is set to *R* = 7000 $, and the variable income coefficient is set to *r* = 1000 $/Mbit. In addition, for the local computing power of the smart terminal *i*, it is set to a value randomly generated from a uniform distribution within GHash/s. Finally, the unit cost of the computing resources of the edge server is set to *p* = 10 $/GHash (that is, the cost of 10 $ is required to complete 1 G hash operations. The specific parameter settings are shown in Table 4.

The variation of the overall net benefit with different *μ* (the total computing power obtained by all smart terminals from the edge server) is shown in Figure 7. The figure shows that when *μ* increases, the overall net benefit first increases, and then when *μ* exceeds a certain threshold, the overall net benefit gradually decreases. This change in overall net income was very well in line with expectations. That is, too small *μ* or too large *μ* will not benefit the offloading of computing tasks. On the one hand, when *μ* is too small, the intelligent terminal can only obtain a small amount of computing power from the edge server. This results in a small overall net benefit. On the other hand, when *μ* is too large, a large cost is incurred for obtaining computing power. This again reduces total net income. This phenomenon is the main part of the work of this chapter. That is, finding the best trade-off between utilizing the computing power provided by edge servers and the consequent cost.

To clarify, all results were obtained on a PC with Intel Core i5-4590 CPU@3.3 GHz. The K-means algorithm can achieve the global optimal solution as a benchmark scheme. Moreover, the K-means algorithm designed in this paper consumes less computation time than the benchmark scheme. Thus, the effectiveness of the algorithm proposed in this paper is verified. The performance test of K-means algorithm is shown in Table 5.

The article "Blockchain and K-Means Algorithm for Edge AI Computing" was retracted in 2023. Reasons: unreliable results or conclusions; concerns about the data; concerns about the results or conclusions; concerns about the peer review.

Figure 8 shows the impact of the edge server providing computing power for intelligent terminals on the cost coefficient *pp*. When the cost coefficient *p* increases, the intelligent terminal becomes conservative when using the computing resources from the edge server. Hence the total computing power obtained from the edge servers is reduced. Similarly, when the cost coefficient *p* increases, the total net benefit of all smart terminals gradually decreases.

It is based on Bandwidth Awareness (BA), the controller of the BA method does not apply any bandwidth allocation strategy. That is, each user node runs Scoot Player. The requested fragment bitrate is based on the player's own bandwidth-aware bitrate selection algorithm. The research environment is shown in Table 6.

It can be seen from Figure 9 that when the number of nodes is greater than 16, the consensus delay of the K-means algorithm based on partition clustering is significantly lower than that of the original K-means algorithm, the OBFT algorithm, and the K-means algorithm based on the scoring and sorting mechanism. Moreover, with the increase in the number of nodes, the delay of the other three algorithms increases greatly. In contrast, the delay of the K-means algorithm based on partition clustering has almost no increase. The improved K-means algorithm based on partition clustering divides nodes into several clusters through cluster analysis. Therefore, the node does not need to communicate with each node, but only needs to communicate with the nodes in the cluster. At the same time, the improved clustering algorithm performs clustering through the number of routes between nodes and the delay between nodes. This reduces the communication delay of nodes within the cluster. The experimental results reflect the role of the improved clustering algorithm in the K-means algorithm. It shows that the K-means algorithm based on partition clustering greatly reduces the consensus delay and increases the consensus efficiency when the number of nodes is large. The algorithm consensus delay comparison is shown in Figure 9.

## 5. Discussion

In a centralized system, the consensus among nodes is achieved by nodes with high decision-making power. Therefore, the more centralized the decision-making power is, the easier it is to reach a consensus. Ethereum currently uses Proof of Work (PoW) as a consensus protocol between nodes. However, this consensus mechanism needs to consume a lot of computing power, resulting in a waste of resources. Therefore, more and more consensus mechanisms have been proposed to solve the problem of consensus among nodes in decentralized systems.

The article "Blockchain and K-Means Algorithm for Edge AI Computing" was retracted in 2023. Reasons: unreliable results or conclusions; concerns about the data; concerns about the results or conclusions; concerns about the peer review.

A blockchain is a chronological connection of blocks containing transaction data. It is a chained data structure composed of hash encryption technology. It is used to record transaction information and data to ensure the security and immutability of transactions in a cryptographic manner. This distributed ledger is stored among all participants in the P2P network. After the participants calculate and obtain the accounting rights, they use encrypted signatures to add the new transaction list to the existing blockchain to form a secure, continuous, and immutable chain data structure. In traditional distributed databases, a centralized third-party server node stores and maintains data, and other nodes save data backups. In the blockchain network, its distributed characteristics are not only reflected in the distributed data storage backup, but also in the distributed data records. That is, all nodes jointly participate in the maintenance of ledger data. Each node has the opportunity to participate in the update of the ledger, but must obtain the consent of the majority of nodes. Therefore, the tampering or destruction of the blockchain data of a few nodes will not affect the content of the transaction ledger stored in the entire blockchain. In this way, secure storage of transaction data is achieved.

By integrating idle computing resources in an area, a distributed edge computing platform is formed. Users obtain benefits by sharing their computing resources, and nodes in need complete computing tasks through the shared platform. Aiming at the identity security problems faced in the sharing process, blockchain technology is introduced to realize the trust between users. All participants must register a secure identity in the blockchain network and conduct transactions in this security system. For mobile edge computing, a large number of computing tasks must involve wireless communication between mobile users and edge clouds. Therefore its performance is highly dependent on wireless access efficiency. Due to the inherent limitations of radio resources, if the wireless access calculation among multiple mobile users is not well coordinated. Then the wireless network capacity may be quickly compressed by the large number of wireless access tasks. This leads to inefficiencies in transmission (long delays in data transmission, and ultimately leads to dissatisfaction with mobile edge computing services.

## 6. Conclusion

Computing offloading provides computing resources for resource-constrained devices to run computing-intensive applications and speeds up computing. While saving energy, it also brings about reliability problems of calculation results. For example, for computations that consume a lot of resources, the remote server may return a result that is not fully computed or an answer that is not computed, to save computing resources. The issue of computational reliability has led to numerous studies of verifiable computation. To solve the problem of result reliability in mobile edge computing offloading, this paper proposes a noninteractive zero-knowledge verifiable computing framework based on blockchain. The framework verifies the calculation results according to the complete trustworthiness of the smart contracts on the blockchain and combines zero-knowledge proofs to ensure the reliability of the calculation results. The prototype of the framework is built, the feasibility of the framework is verified, and the computational consumption and time consumption of the framework are experimentally analyzed. In the follow-up, it is necessary to further study the homomorphic encryption algorithm with better performance or further optimize the consensus algorithm, network propagation method, etc., so as to improve the transaction processing capability of the system.

The article "Blockchain and K-Means Algorithm for Edge AI Computing" was retracted in 2023. Reasons: unreliable results or conclusions; concerns about the data; concerns about the results or conclusions; concerns about the peer review.

## Figures and Tables

**Figure 1:** System model.

**Figure 2:** Structure of a BAcombo node.

**Figure 3:** Energy consumption optimization values of various algorithms under different MEC numbers.

**Figure 4:** Iterative process of the four algorithms.

**Figure 5:** Changes in the number of blocks and the energy consumption of processing data.

**Figure 6:** Latency comparison of different processing schemes.

**Figure 7:** Overall net benefit as a function of *μ* (total computing power obtained by all smart terminals from edge servers).

**Figure 8:** The impact of edge servers providing computing power to intelligent terminals on the cost coefficient *p*.

**Figure 9:** Comparison of algorithm consensus latency.

**Table 1:** Dataset information of 10 blocks (blocks 0–9).

Block number *k*	Timestamp	Block size	Used space	PoW
0	0	540	5	17179869184
1	1438269988	537	10	17171480576
2	1438270017	544	47	171 63096064
3	1438270048	1079	40	171 54715646
4	1438270077	1079	6	17146339321
5	1438270083	537	50	17154711556
6	1438270107	537	41	17146335232
8	1438270110	1078	108	17154707466
9	1438270112	544	10	171 63083788

**Table 2:** Minimum energy consumption comparison of four algorithms.

*N*	SA	GA	ACO	K-means
*n* = 10	108.4	108.4	95.3	88.9
*n* = 50	109.5	109.5	98.1	93.6
*n* = 100	111.2	111.2	99.9	98.5

**Table 3:** Comparison of iteration times of the four algorithms.

*N*	SA	GA	ACO	K-means
*n* = 10	143	73	52	43
*n* = 50	109	59	66	57
*n* = 100	218	90	107	66

**Table 4:** Specific parameter settings.

Significance	Numerical value
The local computing power of the smart terminal *i*	Evenly distributed between 1 and 2 GHash/s
Block size of smart terminal *i*	1 Mbit
Fixed income on blocks	7000$
Variable revenue coefficient of the block	1,000 $/Mbit
Average generation rate per block	1/600
Marginal price of computing power	10 $/GHash

The article "Blockchain and K-Means Algorithm for Edge AI Computing" was retracted in 2023. Reasons: unreliable results or conclusions; concerns about the data; concerns about the results or conclusions; concerns about the peer review.

**Table 5:** Performance testing of K-means algorithm.

5 user scenarios	*t* = 0.2 Mbit	*t* = 0.4 Mbit	*t* = 0.6 Mbit
K-means algorithm results	52.4482	52.6437	52.8338
K-means algorithm consume time	0.314 s	0.278 s	0.249 s
CVX results	52.4482	52.6437	52.8338
CVX consume time	148.5 s	154.4 s	140.39 s

**Table 6:** Research environment.

Bitrate level	Bitrate	Bottleneck bandwidth
0	50	787611
1	200	
2	300	

## Data Availability

No data were used to support this study.
